The article "Prevalence of mycorrhizae in host plants and rhizosphere soil: A biodiversity aspect" was retracted in 2022. Reasons: compromised peer review; a conflict of interest; concerns about the authorship.

# Prevalence of mycorrhizae in host plants and rhizosphere soil: A biodiversity aspect

**DOI:** 10.1371/journal.pone.0266403

**Published:** 2022-03-31

**Authors:** Majidul Islam, Abdulrahman Al-Hashimi, Mosa Ayshasiddeka, Hanif Ali, Hesham Ali El Enshasy, Daniel Joe Dailin, R. Z. Sayyed, Tanzima Yeasmin

**Affiliations:** 1 Department of Biochemistry and Molecular Biology, University of Rajshahi, Rajshahi, Bangladesh; 2 Department of Botany and Microbiology, College of Science, King Saud University, Riyadh, Saudi Arabia; 3 Institute of Bioproduct Development, Universiti Teknologi Malaysia (UTM), Skudai, Johor Bahru, Malaysia; 4 Faculty of Engineering, School of Chemical and Energy Engineering, Universiti Teknologi Malaysia (UTM), Skudai, Johor Bahru, Malaysia; 5 City of Scientific Research and Technology Applications (SRTA), New Burg Al Arab, Alexandria, Egypt; 6 Department of Microbiology, PSGVP Mandal’s S I Patil Arts, G B Patel Science, and STKVS Commerce College, Shahada, India; 7 Department of Entomology, Asian PGPR Society, Aurburn University, AL, United States of America; The University of Haripur, PAKISTAN

## Abstract

Plants roots are colonized by soil inhabitants known as arbuscular mycorrhizal fungi (AMF), which increase plant productivity, and enhance carbon storage in the soil. We found mycorrhizal vesicles, arbuscles, and mycelium in the root of more than 89% of the selected plants of University of Rajshahi campus, Bangladesh. The rate of their presence differed in plant to plant of a family and different families. The highest root colonization (98±1.0%) was found to be present in *Xanthium strumarium* (Asteraceae). Mycorrhiza was not found in the root of *Sphagneticola calendulacea* (Asteraceae), *Cestrun nocturnum* (Solanaceae), *Acacia nilotica* and *Acacia catechu* (Mimosoidae), *Rorippa nasturtium*, *Brassica oleracla var botrytis* (Brasicaceae), *Punica granatum* (Lythraceae), *Tecoma capensis* (Bignoniacea), *Spinacia oleracia* (Chenopodiaceae), *Chenopodium album* (Goosefoot). Result of soil analysis reveals that the rhizospheric soils were deficient in nutrients which might be suitable for mycorrhizal symbiosis with plants. In the rhizospheric soils, 22 species of *Glomus*, *Scutelospora*, *Gigaspora*, *Archaeospora*, *and Acullospora* were found. We also found the genera ’*Glomus*’ dominance in the plant root and rhizospheric soil. So, it can be concluded that the highly colonized roots as well as spores can be used to prepare mycorrhizal inoculum for future purposes.

## Introduction

Arbuscular mycorrhiza (AM) is the plant-fungal symbiosis that exists on the Earth [1,2]. Smith and Read [2] revealed that more than 90% of all plant species, from liverworts to angiosperms are involved in the mycorrhizal association [3]. In some cases, soil pH, soil phosphate (P) level, salinity vegetation, or the hydrologic condition of the soil have been found to be associated with the distribution of AM fungal species [4–7]. A decrease in either AM colonization in roots or the number of fungal propagules in soil was found to be associated with high values of soil pH, nutrient status, moisture content, and salinity [8].

Carbohydrates are produced in the leaves and then transported to the root tissue by the plant’s stomata. Fungal partners in mycorrhizal association obtain carbohydrates from the roots of the host plant. As a result, the fungus has access to a steady supply of glucose and sucrose from the host plants. The fungal hyphae produce large surface area. Compared to plant roots hair, these hairs are much longer and finer. These are capable of releasing minerals from the soils that aren’t accessible to plants roots. However, the fungal partner absorbs water and mineral nutrients from the soil and supplies the plants. Increased plant growth and development in nutrient-poor soil can be achieved as a result of this effect [9].

Economic growth in Bangladesh relies heavily on the production of agricultural crops. Increased production costs and the harmful nature of chemical fertilizers for the environment have sparked renewed interest in the use of less expensive and technologically simple methods for environmental sustainability with low production costs and high crop yields. Various plant species are naturally grown in the Rajshahi University area, Bangladesh. In addition, a wide variety of crops, fruits and vegetables are grown by people. Most of the Rajshahi zone’s plant species are naturally grown on the campus of University of Rajshahi, while others are cultivated. The goal of this investigation was to discover the biodiversity of mycorrhizal organisms in plant roots and rhizospheres. In future, mycorrhizal inoculum will be prepared using highly colonized roots as well as mycorrhizal spores as an alternative to chemical fertilizers by gathering knowledge about the status of biodiversity. As a result, mycorrhizal technology can be used to improve crop yields and environmental quality in Bangladesh’s various agricultural systems.

## Materials and methods

### Study area

The study area, University of Rajshahi, Bangladesh has been selected as representative of Rajshahi Zone, Bangladesh. It is located in the district of Rajshahi and situated at 24.370°N 88.637°E northwestern part of Bangladesh with an area of approximately 753 acres. The altitude of Rajshahi is 30 m.a.s.l. It is on the bank of the river, Padma. The temperature recorded is 26°C to 42°C, and the average rainfall is 280 mm.

### Sample collection

About 91 different plant species were selected randomly (Table 1). The root samples along with rhizospheric soil were collected at a depth of 0–20 cm with the auger. Number of samples for each plant is one for soil sample and root pieces, and three plants are considered for each species.

**Table 1:** Scientific name and family of the selected plants to study the prevalence of mycorrhizae.

Plant Name	Family	Plant Name	Family
*Xanthium Strumarium*	Asteraceae	*Coccinea cordifolia*	Cucurbitaceae
*Chrysanthemum sp*	Asteraceae	*Benincasa hispida*	Cucurbitaceae
*Tagetes Minuta*	Asteraceae	*Gardenia jasminoides*	Rubiaceae
*Eclipta alba*	Asteraceae	*Ixora coccinea*	Rubiaceae
*Mikania scandens*	Asteraceae	*Coffea arabica*	Rubiaceae
*Blumea lacera*	Asteraceae	*Salvia divinorum*	Lamiaceae
*Calendula arvenris*	Asteraceae	*Leonurus sibiricus*	Lamiaceae
*Helianthus annus*	Asteraceae	*Clerodendrum inerme*	Lamiaceae
*Cosmos bipinatus*	Asteraceae	*Ocimum sanctum*	Lamiaceae
*Enhydra fluctuans*	Asteraceae	*Salvia officinalis*	Lamiaceae
*Synedrella nodiflora*	Asteraceae	*Lantana camara*	Verbenaceae
*Sphagneticola calendulacea*	Asteraceae	*Verbena lilacina*	Verbenaceae
*Solanum melongena*	Solanaceae	*Nyctanthes arborstritis*	Oleaceae
*Datura metal*	Solanaceae	*Jasmin sambac*	Oleaceae
*Capsicum frutecens*	Solanaceae	*Rumex maritimus*	Polygonaceae
*Nicotiana plumbagenifolia*	Solanaceae	*Polygonum sp*	Polygonaceae
*Petunia hybrid*	Solanaceae	*Cassia tora*	Cesalpinaceae
*Lycopersicon lycopersicum*	Solanaceae	*Puozologia indica*	Cesalpinaceae
*Solanum indicum*	Solanaceae	*Cassia sophera*	Cesalpinaceae
*Cestrun nocturnum*	Solanaceae	*Lagerstoemia flosreginae*	Lythraceae
*Hibiscus rosa-sinensis*	Malvaceae	*Punica granatum*	Lythraceae
*Abelmoschus esculentus*	Malvaceae	*Bacopa monnieri*	Plantoginaceae
*Sidarhombifolia*	Malvaceae	*Penstemon babatus*	Plantoginaceae
*Sidaacuta*	Malvaceae	*Acacia catechu*	Mimosoidae
*Amaranthus spinosus*	Amaranthaceae	*Acacia nilotica*	Mimosoidae
*Amaranthus viridis*	Amaranthaceae	*Phyllanthus reticulutus*	Phyllanthaceae
*Alternanthera sessilis*	Amaranthaceae	*Phyllanthus fraternus*	Phyllanthaceae
*Alternanthera sp*	Amaranthaceae	*Heliotropium indicum*	Boraginaceae
*Achyranthus aspera*	Amaranthaceae	*Tropaeolum majus*	Tropaeolaceae
*Mimosa pudica*	Fabaceae	*Catharanthus roseus*	
*Sesbania aculiata*	Fabaceae	*Thuja sp*	Cupersaceae
*Peltophorum pterocarpum*	Fabaceae	*Carica papya*	Caricaceae
*Crotalaria sp*	Fabaceae	*Artocarpus heterophyllus*	Moraceae
*Acacia auriculiformis*	Fabaceae	*Impatiens balsamina*	Balsaminaceae
*Delonix regia*	Fabaceae	*Pteris pteris*	Pteridaceae
*Codiaeum varicgatum*	Euphorbiaceae	*Poa annua*	Poaceae
*Acalypha indica*	Euphorbiaceae	*Litchi chinensis*	Sapindaceae
*Euphorbia hypericifolia*	Euphorbiaceae	*Psidium guajava*	Myrtaceae
*Ricinus communis*	Euphorbiaceae	*Murraya paniculata*	Rutaceae
*Ricinus sp*	Euphorbiaceae	*Blubell barleria*	Acanthaceae
*Euphorbia mili*	Euphorbiaceae	*Adhatoda vasica*	Acanthaceae
*Zea mays*	Poaceae	*Rorippa nasturtium*	Brassicaceae
*Triticum aestivum*	Poaceae	*Brassica oleracia var botrytis*	Brassicaceae
*Cynodon dactylon*	Poaceae	*Tecoma capensis*	Bignoniaceae
*Elymus repens*	Poaceae	*Spinacia oleracia*	Chenopodiaceae
*Cucurbita maxima*	Cucurbitaceae	*Chenopodium album*	Goosefoot

### Assessment of root colonization

Fixed root pieces were washed with 70% alcohol and then washed three times with distilled water. After that, root pieces were selected and cut into small segments (about 1 cm). Root segments were put in a beaker containing enough 10% KOH solution, covered, and heated at 90°C in the water bath for 60 min. KOH was poured off and washed with distilled water three times. Root pieces were treated with alkaline H_2_O_2_ for 20 min. at room temperature. Then, these were rinsed with distilled water three times and acidified with 1% HCl for 3 min. Root pieces were stained with trypan blue solution for 120–180 min., and subsequently, the root was de-stained at room temperature in lactoglycerol. After de-staining, these root segments were examined under the microscope to observe mycorrhizal root colonization. The extent of VA mycorrhizal colonization was estimated by the percentage of root length colonization examined for each sample at least 50 root segments [10] and calculated by the following formula–

$$Root\;colonization\;(\%)=\frac{No.\;of\;AM\;positive\;segments}{No.\;of\;segments\;studied}x100$$

#### Extraction, identification, and quantification of mycorrhizal spores

Collected soil samples were dried in the air, and 100 g of air-dried soil sample was taken in a bucket filled with ¾^th^ in tap water and mixed water properly, and left to settle down for about 5–10 min. The supernatant was decanted, and sucrose gradient centrifugation was done for 4 min. at 3000 rpm [11]. Spores were counted under a dissecting microscope, and spore densities (SD) were expressed as the number of spores per 100 g of soil. The isolated spores were mounted in polyvinyl lactoglycerol (PVLG). Morphological identification of spores up to species level was based on spore size, color, the thickness of the wall layers, and the subtending hyphae by the identification manual [http://schuessler.userweb.mwn.de/amphylo] and the website of the international collection of vesicular and AM fungi (http://invam.wvu.edu).

### Soil analysis

Air-dried rhizospheric soil samples in three replicates for each plant were analyzed for their physical and chemical properties. The pH was determined (soil-water suspensions) with the help of a pH meter [12]. The texture was determined using 6% H_2_O_2_, 2N HCl, and 2N NaOH [13]. The moisture content was determined according to the conventional method. Organic matter (OM) was determined by the Walkley-Black acid digestion method. Phosphorus (extracted with 0.03M NH4F-0.02M HCl) was measured by molybdenum blue colorimetry method, potassium (K) by an ammonium acetate method using a flame photometer, and nitrogen (N) by the alkaline hydrolysis diffusion method. Available soil Boron and Zinc were determined in atomic spectrophotometer [14].

### Statistical analysis

All experiments were conducted in triplicate. The data was analyzed by One-way analysis of variance (ANOVA), and the values of standard deviations were considered. The p-value (p < 0.05, < 0.001) was considered in determining significant difference.

## Results

### Presence of AMF structure in roots

The plants of University of Rajshahi showed a well-colonized arbuscular mycorrhizal association. The occurrence of Mycorrhizal fungi in roots of plants has been determined on the basis of vesicles, arbuscular and hyphal formation (Fig 1).

**Fig 1:** (A, B, C, N, S) *Codiaeum varicgatum* (D, E, F) *Salvia divinorum* (G, H, V, X) *Clerodendrum inerme* (I) *Xanthium strumarium* (J) *Phyllanthus reticulutus* (K) *Benincasa hispida* (L) *Eclipta alba* (M) *Salvia officinalis* (O) *Nicotiana plumbaginifolia* (P, Q, R) *Catharanthus roseus* (T) *Phyllanthus reticulutus* (U) *Nyctanthes arborstritis* (W) *Amaranthus viridis* colonized with mycorrhizal arbuscles, vesicles and mycelium externally and internally, magnified at 100X.

### Root colonization in roots of different plants

The percentage of root colonization was compared among 91 different plant species. About 89% of plants were found to be colonized with AMF, and the degree of colonization varied from 10.3±0.6% to 98.0±1.0%, as shown in Table 2. The highest colonization (98±1.0%) was observed in *Xanthium strumarium* belonging to the family Asteraceae. In contrast, other plants of Asteraceae i.e. *Chrysoxanthum* sp, *Tagetes minuta*, *Eclipta alba*, *Mikania scandens*, *Blumea lacera*, *Calendula arvenris*, *Hellianthus annus*, *Cosmos bipinatus*, *Enhydra fluctuans*, and *Synedrella nodiflora* showed root colonization 80.3±2.5%, 75.3±1.5%, 72.7±2.5%, 59.7±2.1%, 48.0±5.0%, 42.3±4.0%, 29.7±0.6%, 24.3±4.0%, 20.3±2.5% and 18.7±4.0% respectively. *Sphagneticola calendulacea* was not colonized with mycorrhiza. The percentage of root colonization varied from 18.7±4.0% to 98±1.0% in the Asteraceae family. In the Solanaceae family, the highest colonization (80.7±3.1%) was observed in *Datura metal*, whereas *Solanum melongena*, *Capsicum frutecens*, *Nicotiana plumbaginifolia*, *Petunia hybrid*, *Lycopersicon lycopersicum*, and *Solanum indicum* showed 80.3±2.5%, 73.3±0.6%, 69.0±4.6%, 51.0±3.6%, 49.7±3.8% and 34.0±3.6% respectively. The percentage colonization ranged from 34.0±3.6% to 80.7±3.1% in the Solanaceae family. No colonization was observed in *Cestrun nocturnum*. In the Malvaceae family, highest (59.3±4.0%) and lowest (11.3±1.2%) colonization was observed in *Hibiscus rosa-sinensis and Sida acuta*, respectively, whereas *Abelmoshcus esculentus* and *Sida rhombifolia* showed 52.3±3.5% and 31.7±1.5% individually. The percentage of root colonization speckled from 11.3±1.2% to 59.3±4.0% in the Malvaceae family. Among five plants of the Amaranthaceae family, the highest colonization (75.3±2.5%) was found in *Amaranthus spinosus*, and *Alternanthera* sp. showed the lowest colonization (11.0±1.7%), whereas *Achyranthus aspera*, *Alternanthera sessilis*, *and Amaranthus viridis* showed 11.3±1.5%, 21.3±3.2%, and 39.7±2.5% root colonization respectively. The root colonization varied from 11.0±1.7% to75.3±2.5% in the Amaranthaceae family. In the Fabaceae family, the highest colonization (35.7±2.1%) was observed in *Mimosa pudica*, whereas *Sesbania aculiata*, *Peltophorum pterocarpum*, *Crotalaria* sp. *Acacia auriculiformis*, *and Delonix regia* showed 33.0±2.6%, 30.7±2.1%, 21.0±5.6%, 16.0±3.6%, and 11.0±1.7% respectively. The percentage colonization ranged from 11.0±1.7% to 35.7±2.1% in the Fabaceae family. In the Acanthaceae family, the highest colonization (42.3±8.5%) was observed in *Blubell barleria*, whereas *Adhatoda vasica* showed 33.7±9.5% root colonization. In the Euphorbiaceae family, the highest colonization (90.3±2.5%) was found in *Codiaeum varicgatum*, and *Euphorbia mili* showed the lowest colonization (10.7±1.2%). Other plants of this Family i.e. *Acalypha indica*, *Euphorbia hypericifolia*, *Ricimus* sp., *and Ricinus communis* showed 41.3±4.2%, 37.7±3.5%, 25.3±0.6, and 19.3±2.1 respectively. The mycorrhizal colonization ranged from 10.7±1.2% to90.3±2.5% in the Euphorbiaceae family. In the Poaceae family, the highest colonization (49.0±3.6%) was detected in *Zea mays*. Other plants of this family i.e. *Triticum aestivum*, *Cynodon dactylon*, and *Elymus repens* showed 29.7±0.6%, 15.3±1.5%, and 11.7±1.5% separately. The root colonization varied from 11.7±1.5% to 48.0±2.0% in the Poaceae family. In the Cucurbitaceae family, the highest root colonization (80.3±2.1%) was found in *Cucurbita maxima*. Other plants of this family i.e. *Coccinea cordifolia*, *Benincasa hispida* showed 44.3±3.1, and 40.7±2.1% respectively. The percentage of root colonization varied from 40.7±2.1% to 80.3±2.1% in the Cucurbitaceae family. Among the plants of the Rubiaceae family, the highest root colonization (50.0±2.6%) was detected in *Ixora coccinea and Gardenia jasminoides*, *Coffea arabica* showed 10.7±1.2%, 40.0±2.0% root colonization respectively. The percentage of root colonization varied 10.7±1.2% to 50.0±2.6% in the Rubiaceae family. In the Lamiaceae family, *Salvia divinorum*, *Clerodendrum inerme* showed a maximum of 85.7±1.2%, 85.7±2.1% respectively. Other plants of this family i.e. *Leonurus sibiricus*, *Ocimum sanctum*, *Salvia officinalis* showed 85.0±4.0%, 38.3±5.5%, 32.3±6.7% root colonization respectively. The percentage of root colonization varied 32.3±3.1% to 85.7±1.2% in the Lamiaceae family. In the Oleaceae family, *Nyctanthes arborstritis* showed the highest root colonization (66.0±4.6%), whereas *Jasmin sambac* showed 40.0±7.0% root colonization. In the Polygonaceae family, *Polygonum* sp. showed 36.7±5.5% root colonization, where *Rumax maritimus* showed 11.0±1.0% mycorrhizal root colonization. In the Caesalpinaceae family, *Cassia tora*, *Puozolgia indica*, *and Cassia sophera* showed 59.7±8.5%, 25.0±3.6%, and 26.7±3.8% mycorrhizal root colonization respectively. In the Lythraceae family, *Lagerstroemia flosregia* showed 41.7±7.5% root colonization, whereas *Punica granatum* did not show mycorrhizal root colonization. In the Plantaginaceae family, *Bacopa monnieri* and *Penstemon babatus* showed 30.0±7.0%, 30.7±3.1% mycorrhizal root colonization separately. *Phyllanthus reticulutus (Phyllanthaceae)*, *Tropaeolum majus* (Tropaeolaceae), *Heliotropium indicum* (Boraginaceae), *Catharanthus roseus* (Apocynaceae), *Thuja* sp. (Cupresaceae), *Carica papya* (Caricaceae), *Artocarpus heterophyllus* (Moraceae), *Impatiens balsamina* (Balsaminaceae) *and Pteris pteris* (Pteridaceae) showed 74.3±1.5%, 46.3±5.5%, 46.0±2.0%, 44.7±2.5%, 38.3±5.1%, 34.3±1.2%, 30.7±8.0%, 25.0±2.6% and 19.7±6.5% respectively. *Poa annua* (Grass), *Litchi chinensis* (Sapindaceae), *Psidium guajava* (Myrtaceae), and *Murraya paniculata* (Rutaceae) showed 11.7±1.5%, 10.3±0.6%, 12.3±2.5%, 13.0±3.6% root colonization separately. *Acacia nilotica and acacia catechu* (Mimosoideae), *Calotropis procera* (Asclepiadaceae), *Rorippan asturtium* (Brassicaceae), *Tecoma capensis* (Bignoniaceae), *Spinacia oleracia* (Chenopodiaceae), *Chenopodium album* (Groosefoot) did not show mycorrhizal root colonization.

**Table 2:** Mycorrhizal root colonization in different plants of Rajshahi University campus ground.

Plant Name	Family	Root colonization	Scientific Name	Family	Root colonization
*Xanthium Strumarium*	Asteraceae	98.0±1.0	*Coccinea cordifolia*	Cucurbitaceae	44.3±3.1
*Chrysanthemum* sp.	Asteraceae	80.3±2.5	*Benincasa hispida*	Cucurbitaceae	40.7±2.1
*Tagetes Minuta*	Asteraceae	75.3±1.5	*Gardenia jasminoides*	Rubiaceae	10.7±1.2
*Eclipta alba*	Asteraceae	72.7±2.5	*Ixora coccinea*	Rubiaceae	50.0±2.6
*Mikania scandens*	Asteraceae	59.0±3.6	*Coffea arabica*	Rubiaceae	40.0±2.0
*Blumea lacera*	Asteraceae	48.0±5.0	*Salvia divinorum*	Lamiaceae	85.7±1.2
*Calendula arvenris*	Asteraceae	42.3±4.0	*Leonurus sibiricus*	Lamiaceae	85.0±4.0
*Helianthus annus*	Asteraceae	29.7±0.6	*Clerodendrum inerme*	Lamiaceae	85.7±2.1
*Cosmos bipinatus*	Asteraceae	24.3±4.0	*Ocimum sanctum*	Lamiaceae	38.3±5.5
*Enhydra fluctuans*	Asteraceae	20.3±2.5	*Salvia officinalis*	Lamiaceae	32.3±6.7
*Synedrella nodiflora*	Asteraceae	18.7±4.0	*Lantana camara*	Verbenaceae	36.3±4.2
*Sphagneticola calendulacea*	Asteraceae	0	*Verbena lilacina*	Verbenaceae	28.7±5.0
*Solanum melongena*	Solanaceae	80.3±2.5	*Nyctanthes arborstritis*	Oleaceae	66.0±4.6
*Datura metal*	Solanaceae	80.7±3.1	*Jasmin sambac*	Oleaceae	40.0±7.0
*Capsicum frutecens*	Solanaceae	73.3±0.6	*Rumex maritimus*	Polygonaceae	11.0±1.0
*Nicotiana plumbagenifolia*	Solanaceae	69.0±4.6	*Polygonum* sp.	Polygonaceae	36.7±5.5
*Petunia hybrid*	Solanaceae	51.0±3.6	*Cassia tora*	Cesalpinaceae	59.7±8.5
*Lycopersicon lycopersicum*	Solanaceae	49.7±3.8	*Puozologia indica*	Cesalpinaceae	25.0±3.6
*Solanum indicum*	Solanaceae	34.0±3.6	*Cassia sophera*	Cesalpinaceae	26.7±3.8
*Cestrun nocturnum*	Solanaceae	0	*Lagerstoemia flos reginae*	Lythraceae	41.7±7.5
*Hibiscus rosa-sinensis*	Malvaceae	59.3±4.0	*Punica granatum*	Lythraceae	0
*Abelmoschus esculentus*	Malvaceae	52.3±3.5	*Bacopa monnieri*	Plantoginaceae	30.0±7.0
*Sidarhombifolia*	Malvaceae	31.7±1.5	*Penstemon babatus*	Plantoginaceae	30.7±3.1
*Sidaacuta*	Malvaceae	11.3±1.2	*Acacia catechu*	Mimosoidae	0
*Amaranthus spinosus*	Amaranthaceae	75.3±2.5	*Acacia nilotica*	Mimosoidae	0
*Amaranthus viridis*	Amaranthaceae	39.7±2.5	*Phyllanthus reticulutus*	Phyllanthaceae	74.3±1.5
*Alternanthera sessilis*	Amaranthaceae	21.3±3.2	*Phyllanthus fraternus*	Phyllanthaceae	19.7±3.8
*Alternanthera* sp.	Amaranthaceae	11.0±1.7	*Heliotropium indicum*	Boraginaceae	46.0±2.0
*Achyranthus aspera*	Amaranthaceae	11.3±1.5	*Tropaeolum majus*	Tropaeolaceae	46.3±5.5
*Mimosa pudica*	Fabaceae	35.7±2.1	*Catharanthus roseus*		44.7±2.5
*Sesbaniaaculiata*	Fabaceae	33.0±2.6	*Thuja* sp.	Cupersaceae	38.3±5.1
*Peltophorum pterocarpum*	Fabaceae	30.7±2.1	*Carica papya*	Caricaceae	34.3±1.2
*Crotalaria* sp.	Fabaceae	21.0±5.6	*Artocarpus heterophyllus*	Moraceae	30.7±8.0
*Acacia auriculiformis*	Fabaceae	16.0±3.6	*Impatiens balsamina*	Balsaminaceae	25.0±2.6
*Delonix regia*	Fabaceae	11.0±1.7	*Pteris pteris*	Pteridaceae	19.7±6.5
*Codiaeum varicgatum*	Euphorbiaceae	90.7±4.0	*Poa annua*	Poaceae	11.7±1.5
*Acalypha indica*	Euphorbiaceae	41.3±4.2	*Litchi chinensis*	Sapindaceae	10.3±0.6
*Euphorbia hypericifolia*	Euphorbiaceae	37.7±3.5	*Psidium guajava*	Myrtaceae	12.3±2.5
*Ricinus communis*	Euphorbiaceae	19.3±2.1	*Murraya paniculata*	Rutaceae	13.0±3.6
*Ricinus* sp.	Euphorbiaceae	25.3±0.6	*Blubell barleria*	Acanthaceae	42.3±8.5
*Euphorbia mili*	Euphorbiaceae	10.7±1.2	*Adhatoda vasica*	Acanthaceae	33.7±9.5
*Zea mays*	Poaceae	49.0±3.6	*Rorippa nasturtium*	Brassicaceae	0
*Triticum aestivum*	Poaceae	29.7±0.6	*Brassica oleracia var botrytis*	Brassicaceae	0
*Cynodon dactylon*	Poaceae	15.3±1.5	*Tecoma capensis*	Bignoniaceae	0
*Elymus repens*	Poaceae	11.7±1.5	*Spinacia oleracia*	Chenopodiaceae	0
*Cucurbita maxima*	Cucurbitaceae	80.3±2.1	*Chenopodium album*	Goosefoot	0

Values are the average of triplicates. ± indicate standard deviation.

### Physio-chemical properties of rhizosphere soil

The degree to which mycorrhizal fungi enhance the nutrition and health of associated plants depends on many biotic and abiotic soil factors and other environmental factors that influence the host, the fungi, and their association. The most important factors include the abundance of AMF infective propagules and soil phosphorus status. To evaluate higher root colonization against soil chemicals, 8 different plant species i.e. 1 (*Codiaeum varicgatum*), 2 (*Salvia divinorum*), 3 (*Solanum melongena*), 4 (*Tagetes minuta*), 5 (*Phyllanthus reticulutus*), 6 (*Capsicum frutecens*), 7 (*Lycopersicon lycopersicm*), and 8 (*Abelmoshcus esculentus*) were selected for soil analysis. Table 3 summarized the data on soil status, i.e. the physical and chemical properties. It may be mentioned that the status of soil means the suitability of soil conditions for various crop production.

**Table 3:** Physical and chemical parameters of experimental soils, root colonization, and spore number.

	*Codiaeum varicgatum*	*Salvia divinorum*	*Solanum melongena*	*Tagetes minuta*	*Phyllanthus reticulutus*	*Capsicum frutecens*	*Lycopersicon lycopersicm*	*Abelmoshcus esculentus*
Moisture (%)	19.1±0.76	18.3±0.32	18.0±0.26	17.6±0.31	17.3±0.20	17.1±0.29	49.7±3.80	15.5±0.45
pH	8.10±0.20	7.90±0.05	7.90±0.07	7.90±0.06	7.80±0.04	7.80±0.09	7.60±0.11	7.30±0.13
Clay (%)	18.1±0.31	16.5±0.25	15.2±0.35	15.0±0.15	12.0±0.26	10.0±0.44	10.0±0.25	8.00±0.15
Sand (%)	43.33±2.11	47.81±1.03	47.55±0.49	51.72±1.59	55.05±1.10	61.07±1.40	61.80±0.98	64.82±2.06
Silt (%)	38.0±0.32	36.0±0.15	37.5±0.35	33.0±0.25	32.4±0.45	29.0±0.10	29.0±0.38	27.8±0.51
P (ppm)	49.11±0.34	43.81±0.88	36.18±0.44	25.85±1.07	15.48±0.51	57.65±0.92	100.60±1.02	125.19±2.62
N (%)	0.12±0.03	0.10±0.02	0.10±0.03	0.09±0.03	0.08±0.02	0.11±0.01	0.09±0.01	0.10±0.02
C (%)	2.11±0.08	1.71±0.09	1.60±0.07	1.39±0.05	1.81±0.10	1.70±0.12	1.80±0.18	1.70±0.17
K (cmol/kg)	0.32±0.02	0.41±0.03	0.26±0.04	0.16±0.02	0.21±0.05	0.16±0.04	0.17±0.06	1.09±0.09
Zn (ppm)	3.32±0.11	5.89±0.12	4.97±0.14	3.41±0.04	2.28±0.06	7.65±0.24	7.42±0.22	7.38±0.09
B (ppm)	0.76±0.05	1.17±0.03	0.80±0.08	0.55±0.09	0.74±0.08	1.21±0.07	0.64±0.06	1.61±0.18
Colonization	90.3±2.50	85.7±1.20	80.3±2.50	75.3±1.50	74.3±1.50	73.3±0.60	49.7±3.80	52.3±3.50
Spore No.	60.7±1.20	57.7±0.50	50.3±2.10	46.7±2.90	44.0±2.40	35.7±1.70	33.7±2.50	28.7±1.70

Values are the average of triplicates. ± indicate standard deviation.

Soil quality influences mycorrhizal infection. Soil texture may affect plant responses to mycorrhizae. Soil strength and penetration resistance influence the rates at which water and nutrients flow or diffuse to the root surface. The clay, silt, and sand in experimental soils were varied from 8.00±0.15% to 18.1±0.31%, 27.8±0.51% to 38.0±0.32%, and 43.33±2.11% to 64.82±2.06% respectively. So, the observed soils were loamy soil. Loamy soil is suitable for growing most plant varieties.

It was revealed from the present data that the soil pH of the experimental plant area was alkaline, which might be associated with the natural colonization of an arbuscular mycorrhizal fungus in the roots of the plants examined. The pH range was indicated 7.30±0.13 to 8.10±0.20. Khan et al. (2004) reported that the soil pH of the Rajshahi region is high because of naturally alkaline, which is associated with occurring lime [15]. Soil pH is a commonly used index of plant root zone acidity and is crucial to many elements and microbial processes. Moisture influences soil resistance to root penetration, the geometry of different parts of the nutritional movement to root surface, and microorganism activity. The amount of moisture in soil was found to be 15.5±0.45% to 19.1±0.76% in Table 3. Phosphorus is one of the major nutrients for plant growth. It is the structural constituent of nucleotide, which is an energy carrier for all metabolic activities. It is essential for the constituent of the cell nucleus, cell division, and the development of meristematic tissue in the growing regions. The amount of phosphorus in experimental mycorrhizal soils was 15.48±0.51 ppm to 125.19±2.62 ppm. Nitrogen is an essential constituent of protein and, therefore, a constituent of all living cells. Nitrogen increases the proportion of water, and it also makes more giant cells with thinner cell walls.

Nitrogen is an essential constituent of protein and, therefore, a constituent of all living cells. Nitrogen increases the proportion of water, and it also makes more giant cells with thinner cell walls. Soil Nitrogen content was varied from 0.08±0.02 to 0.12±0.03%. Soil organic matter ranged from 1.39±0.05% to 2.11±0.08%. Potassium helps maintain cell permeability, aids in the translocation and composition of carbohydrates, and is essential for photosynthesis. Potassium keeps iron more mobile and increases the resistance of plants to a particular disease. The potassium levels of mycorrhizal rhizosphere soil were ranged between 0.16±0.02 cmol/kg to 1.09±0.09 cmol/kg. Zinc plays a central role in healthy plant metabolism and growth processes. It is needed in small quantities for the formation of auxin, chlorophyll, and cytochrome. It also has a role in forming enzymes and carbohydrates, regulating starches, and proper root development.

Zinc also helps plants assimilate to cold temperatures across the growing season. Zinc plays an essential role in mycorrhizal colonization and distribution. The level of zinc of mycorrhizal rhizosphere soil ranged from 2.28±0.06 ppm to 7.65±0.24 ppm. Boron plays a vital role in a diverse range of plant functions, including cell wall formation and stability, maintenance of structural and functional integrity of biological membranes, movement of sugar or energy into growing parts of plants, and pollination and seed set. Adequate Boron is also required for effective nitrogen fixation and nodulation in legume crops. Boron deficiency commonly results in empty pollen grains, poor pollen vitality, and fewer flowers per plant. Boron has a vital role in colonizing roots with mycorrhizal fungi, which contributes to root uptake of P. The Boron levels of mycorrhizal rhizosphere soil varied from 0.55±0.09 ppm to 1.61±0.18 ppm.

Results showed that mycorrhizal root colonization is positively correlated with number of spores. Correlation among mycorrhizal root colonization, spore numbers, and physiochemical properties of rhizospheric soils of 8 different plant species were summarized in Table 4.

**Table 4:** Pearson correlation among mycorrhizal root colonization, spore numbers, and physiochemical properties of rhizosphere soils of different plant species.

	Colonization	Spore no.	Moisture (%)	Clay (%)	Sand (%)	Silt (%)	pH	P (ppm)	N (%)	C (%)	Zn (ppm)	B (ppm)	K (Cmol/kg)
Colonization	1												
Spore No.	0.915	1											
Moisture (%)	0.954	0.961	1										
Clay (%)	0.983	0.973	0.979	1									
Sand (%)	-0.898	-0.981	-0.952	-0.956	1								
Silt (%)	0.864	0.954	0.918	0.924	-0.986	1							
pH	0.989	0.917	0.943	0.978	-0.884	0.862	1						
P (ppm)	-0.785	-0.673	-0.731	-0.751	0.687	-0.638	-0.738	1					
N (%)	0.437	0.336	0.450	0.403	-0.308	0.328	0.475	0.122	1				
C (%)	0.175	0.263	0.282	0.222	-0.198	0.213	0.243	0.163	0.483	1			
Zn (ppm)	-0.597	-0.621	-0.597	-0.620	0.660	-0.611	-0.535	0.785	0.304	-0.108	1		
B (ppm)	-0.249	-0.387	-0.443	-0.322	0.452	-0.403	-0.180	0.562	0.308	0.019	0.612	1	
K (Cmol/kg)	-0.387	-0.351	-0.511	-0.385	0.362	-0.307	-0.348	0.659	0.020	0.049	0.356	0.805	1

### Mycorrhizal spore density and diversity

The rhizospheric soils which were analyzed to determine physio-chemical properties were selected for isolation of mycorrhizal spores. Twenty-two different mycorrhizal spore populations were isolated. Nineteen isolated spores were identified based on morphological characteristics such as spore size, color, wall thickness, number of walls, types of walls and wall groupings, etc. Three spores could not be identified, which will be identified in future with 18s RNA technology. Identified spores belonged to the genera *Glomus*, *Scutellospora*, *Gigaspora*, *Archaeospora* and *Acullospora* mentioned in Fig 2.

**Fig 2:** Mycorrhizal spores observed in the rhizosphere of different plant species. (A, J) *Acullospora* sp. (B) *Glomus australe* (C, D, G, I, K, O) *Glomus sp* (E) *Gigaspora sp* (F) Unidentified (H) Fossil *gloremycotan* spore L) Unidentified (M) *Archaeospora leptotica* (N) *Glomus fulvum* (P) *Glomus mosseae* (Q) *Gigaspora* sp. (R) *Gigaspora* sp. (S, T) *Scutellospora* sp. (U) Unidentified (V) Sporocarp of *Glomus sinusum*. All spores are 50 μm in size and magnified at 50X.

Isolated spores were varied from 28.7±1.70 to 60.7±1.20 in number per 100 g of soil, as presented in Table 3. The highest spore number was observed in *Codiaeum varicgatum*, while that was lowest in *Abelmoshcus esculentus*.

## Discussion

The study area, University of Rajshahi, Bangladesh has a tropical monsoon climate characterized by heavy seasonal rainfall, high temperatures, and high humidity. The mycorrhizal fungi were found to be present in nearly all of the tested plant species. The intensity varied in the plants of the same family and the plants of different families. Strzemska *et al*. [15] found that the root colonization in the plants of different families and the single-family plants differed [15]. The AM fungal structure in the root varied in the selected plants where vesicles, arbuscles, mycelium were present separately and in combination (Fig 1). Different vesicles were observed where some are oval and some are spherical in shape. Mycelia were present in most of the plants while arbuscles were observed in the roots of some plant species. The observed AMF structure was supported by Khanam *et al*. [16,17]. The frequent occurrence of vesicles in most plant species from the study sites showed the presence of VAM fungi belonging to the *Glomineae*. Plants of Brassicaceae Bignoniaceae, Goosefoot, and Chenopodiaceae were not colonized with mycorrhiza. These data are in line with earlier studies showing that these families lack functional mycorrhizae because of the presence of glucosinolates and their hydrolysis products, isothiocyanates, in and around their roots [18].

In rhizosphere of 8 different plant species, twenty two spores were isolated and nineteen spores were identified as species of *Glomus*, *Scutelospora*, *Gigaspora*, *Archaeospora*, and *Acullospora* (Fig 2) while three spores could not be identified. Among the identified genera, *Glomus* species was found more in number (Ten in twenty-two). Sporocarp of *Glomus sinusum* was observed which indicates that *Glomus* spores are grown in clusters. It might be a reason for getting more number of *Glomus* spores in the roots as shown in Fig 1. *Glomus* is the most common mycorrhizal species in Bangladesh’s forests [19]. They speculated that *Glomus*’ sporulation pattern could be the key to the taxon’s rise to dominance. We found that the rhizosphere and roots of the same plant were found to contain a variety of species from different genera (Figs 1 and 2). Plant phenology, root phenology, and root production all influence spore production patterns [20]. Every life history of a mycorrhizal fungus is influenced by plant roots. Spore germination, germination rate, the direction of germ tubes, hyphal branching recognition of the host root penetration establishment, intensity of colonization growth of hyphae into soils, and sporulation of the AM fungi were reported to be affected by the plant roots [21]. The roots of various plants produced a variety of organic chemicals and volatile compounds. Organic acids, ethanol and other volatile compounds could all influence the AM fungi’s activity and life cycle in natural environments. Various factors, such as dense root systems with an abundance of fine roots, mycorrhizal fungi’s ability to compete with other rhizosphere-dwelling organisms, seasons, soil moisture, soil type, and nutrient levels, have been found to have an impact on spore numbers, activity, and other traits [21].

AM fungal spore number was found to be increased with increase in root colonization. This result is consistent with those of the previous reports [22,23]. However, Fontenla et al. [24] have demonstrated that when the number of spores was high, the frequency of colonization decreased [24]. It has been shown that there is no significant relationship between AM colonization and spore population [25]. It might be due to the different gradients by soil and the strong effect of plant factors on the formation, function, and adaptation of the fungus to the respective soil conditions. Mycorrhizal colonization was found to be possible due to the presence of moisture [26]. Roots were found to have arbuscles when examined under a microscope. Moisture may be a factor for the occurrence of arbuscles. There are several factors that can influence the growth, sporulation, and community structure of AM fungi in the soil [27,28]. The alkaline soil in the experimental area could be linked to the natural colonization of AM fungi [26]. The extraradical proliferation of hyphae may be aided by organic matter, which increases spore production [29,30]. A high level of soil phosphorus generally inhibits mycorrhizal infection [31–34] which might be the reason for current prevalence of mycorrhiza in *Abelmoshcus esculentus*. The potassium concentration might be suitable for mycorrhizal colonization in Bangladesh [35]. The zinc concentration in the soil might be suitable for mycorrhizal root colonization [36]. Mycorrhizal root colonization also affects the zinc nutrition of the crop [37] and is inurn affected by zinc status of the soil [38], climate changes [39,40] and the presence of organic fertilizers and rhizobia [41,42].

However, chemical analysis showed that the rhizospheric soils were deficient in nutrients, especially C, N. Nutrient deficiency might be responsible for the variation in their pattern of production and colonization. By considering all the facts mentioned above, it can be said that the ecological condition of the study area favored diverse mycorrhizal prevalence and their colonization in plant roots.

## Conclusion

This study reveals that in University of Rajshahi, Bangladesh, plant species respond to mycorrhizal association where about 89% plant species are involved in mycorrhizal association. Species of *Acaulospora*, *Gigaspora*, *Glomus*, *Scutelospora*, and *Archaeospora* was observed in the selected rhizospheric soils. Three spores could not be identified which will be confirmed with 18s RNA technology. So, it can be concluded that the highly colonized roots as well as spores can be used in inoculum production on crop of Bangladesh.
